# The Effect on Quality of Life after Three-Dimensional Intensity-Modulated Radiation Therapy in Patients with Low-Grade Glioma

**DOI:** 10.1155/2022/5854013

**Published:** 2022-08-13

**Authors:** Huili Chen, He Rao, Yong Huang

**Affiliations:** Department of Head and Neck Breast Chemoradiotherapy, Zhongnan Hospital of Wuhan University, Hubei Province 430071, China

## Abstract

**Objective:**

To investigate the effect of three-dimensional intensity-modulated radiation therapy (IMRT) that accurately target delineation on quality of life (Qol) in patients with low-grade gliomas.

**Methods:**

From February 2015 to December 2019, 100 patients with low-grade gliomas were randomly divided into three-dimensional conformal radiotherapy control group (*n* = 50) and three-dimensional IMRT research group (*n* = 50). The scores of the Mini-Cog Assessment (Mini-Cog) and Montreal Cognitive Assessment Scale (MoCA), the self-care ability score (BI), and the effect of symptom improvement and the quality of life SF-36 score were compared between the two groups.

**Results:**

After radiotherapy, the self-care ability of patients in the two groups was significantly improved, and the improvement of study group was better than that of the control group (*P* < 0.05). The Mini-Cog and MOCA scores in the study group were significantly higher than those in the control group (*P* < 0.05). In addition, the symptom improvement effect and quality of life of the patients in the study group were also significantly better than those in the control group (*P* < 0.05). The scores of SDS and SAS of patients who underwent three-dimensional conformal IMRT were significantly lower than those of the control group. There was no significant difference in mortality between the two groups.

**Conclusion:**

Three-dimensional conformal intensity-modulated radiation therapy can delineate the target volume more accurately, regulate the intensity of radiation, and improve the symptoms and quality of life of patients with low-grade gliomas.

## 1. Introduction

Glioma is the most common primary brain tumor in adults. WHO classifies glioma into four grades, and clinically, gliomas of grades I to II are called low-grade gliomas (LGG), including low-grade malignant astrocytoma, oligodendrogliomas, and mixed gliomas [1, 2]. The clinical course of LGG is generally less aggressive than that of primary glioblastoma, with its incidence peaking in the third and fourth decade of life [3]. The natural history of tumors is largely determined by the tumor's histological subtype and genetic characteristics. Many patients live 15 years or more, while others die from the disease within a few years. Therefore, individualizing treatment remains a challenge.

Surgery is usually the preferred treatment. Although some patients can be cured, there are still some patients with postoperative recurrence, or most tumors cannot be completely resected due to the limitation of the principle of tumor location and maximum protection of neurological function, and it is easy to transform from low-grade glioma to high-grade glioma [4]. Therefore, in addition to surgical resection, a variety of adjuvant treatments are also required, such as postoperative observation, radiotherapy, chemotherapy, and comprehensive treatment [5]. Adjuvant radiation therapy, as one of the current standard treatment options, has negative short- and long-term impacts on patients' neurocognitive function and health-related quality of life [6]. Three-dimensional conformal radiotherapy is a relatively advanced radiotherapy method, which focuses the radiation on the target area of the tumor according to the main shape of the tumor, so as to avoid unnecessary radiation to the surrounding normal tissues and organs, thus reducing the complications of radiotherapy. Studies [7] have shown that, compared with low dose radiotherapy (45.0 Gy), higher dose radiotherapy (59.4 Gy) has a negative impact on LGG patients' quality of life in the short term. Since patients with low-grade glioma have a longer survival time than patients with high-grade glioma, the choice of treatment should take into account the quality of life of patients, so the relevant follow-up adjuvant radiotherapy has always been a controversial issue. In addition, due to the existence of edema area and the changes of normal anatomical structure after surgery, there are generally large errors in the determination of the target volume of postoperative radiotherapy, especially the definition of clinic target volume (CTV). In recent years, intensity-modulated radiation therapy (IMRT) has been favored because of its better conformity to the radiotherapy target volume and uniform dose distribution, which can better protect normal tissues around the target volume while treating tumors [8, 9]. Due to traumatic brain anatomical site of the specific tumor, with the brain tissue damage of tumor patients, the cognitive function, behavior, and ability are gradually decreased. In addition, radiation therapy is harmful to patients, and radiation damages brain and cognitive function, resulting in pain, severe helplessness, and despair of glioma patients, causing serious damage to their society and family, and even leading to rest and abandonment of treatment. So glioma patients have very low subjective experience of quality of life. With the development of modern medicine, clinical treatment is no longer limited to improving the survival rate and prolonging the survival period, meeting the physiological and psychological needs of postoperative patients, reducing functional sequelae, and improving the quality of life which has become a new trend in clinical research [10, 11]. With the development of the medical model to the biological, psychological, and social medical model, the evaluation index of treatment effect is no longer the single survival time as the only standard, and how to relieve patients' pain and symptoms and improve patients' psychological and life quality has become an important research topic. In the current patient-centered medical situation, efforts to maintain an acceptable quality of life for patients have become the primary goal of cancer treatment, and it is also a secondary indicator of most clinical oncology interventions. Therefore, in this study, 100 patients with low-grade glioma were selected as experimental subjects to explore the impact of IMRT on patients' quality of life.

## 2. Materials and Methods

### 2.1. General Information

In this study, 100 patients with low-grade glioma admitted to our hospital from February 2015 to December 2019 were selected as the research subjects. The average age of patients in the control group was 34.06 ± 5.81 years and a male to female ratio of 15 : 12. The average age of patients in the research group was 38.63 ± 8.21 years and a male to female ratio of 12 : 15. There were no significantly different (*P* > 0.05; Table 1). They were randomly divided into two groups by random number table method, with 50 patients in each group. Inclusion criteria are as follows: (1) patients with clinically diagnosed low-grade glioma according to the guideline for diagnosis and treatment of glioma of central nervous system in China (2015); (2) normal blood routine, biochemical, electrocardiogram, chest X-ray, and abdominal color Doppler ultrasound results before treatment; (3) no lesions in the brain stem; and (4) both patients had clear consciousness and clear complaints before and after treatment. Exclusion criteria are as follows: (1) patients with mental disorders, (2) patients with other tumors, and (3) patients with allergic constitution. This study passed the ethical review of our hospital on January 5, 2015. Before enrollment, we informed patients of the purpose and process of the experiment, obtained informed consent from patients, and signed informed consent.

### 2.2. Research Methods

The control group received conventional three-dimensional conformal radiotherapy. According to the patient's condition, 5-7 irradiation fields were selected for irradiation. The area of glioma expanded by 2 cm was selected as CTV, and the radiation dose for the radical target volume was 66 to 72 Gy, with a total of 33 to 36 times. After operation, the radiotherapy dose for low-risk target volume was 50~54 Gy, with a total of 25~27 times. The radiotherapy dose of high-risk target volume was 56~60 Gy, with 28~30 times in total, once a day, with separated irradiation, 5 times for each week.

In the research group, three-dimensional conformal IMRT was used, and the radiation dose of each site should be controlled. The target volumes of the brain, face, lower neck, and supraclavicular region should be irradiated in a targeted manner. During radiotherapy, the thermoplastic mask was used for fixation, and thin layer (2-3 mm) CT scan was performed with a mesh head frame. CT data were transmitted to Peacock workstation to delineate target volumes and important anatomical structures. According to the location of lesions, the positional relationship between nerves and blood vessels, the tumor volume of patients, the total treatment dose, and the treatment times of patients were input into the workstation for reverse calculation. 80% to 90% were wrapped around the tumor or within the range of 1-2 cm outside the tumor with an isodose curve, and 4-21 treatments were performed with a single dose of 2.5-8 Gy, 3-5 times per week. Both groups of patients were treated with mannitol and hormone therapy after radiotherapy to reduce radiation nerve damage.

### 2.3. Observation Indicators and Curative Effect Standards

(1) The cognitive function of the two groups of patients was analyzed by the Mini-Cog Assessment (Mini-Cog) and the Montreal Cognitive Assessment (MoCA). The Mini-Cog consisted of three-item recall and clock drawing from the Cognitive Abilities Screening Instrument (CASI). In three-item recall, 3 points were calculated for the immediate recall and 3 points for the short-term delayed recall. In clock drawing, a 3-point approach was applied for scoring: 1 point for drawing a circle, 1 point for drawing correct clock numbers, and 1 point for drawing precise clock period. Regular clock drawing was measured when all time criterions were precise, and the hand point was reliable with the indicated time. The MoCA evaluation indexes included executive and visual-spatial function, attention, naming, abstract thinking, linguistic expression, delayed recall, and orientation, with a total score of 0 to 30 points. The higher the score, the better the cognitive function. All the above tests were performed by the same attending physician with relevant training when the patient's mood was stable. (2) Barthel Index (BI) was used to compare patients' self-care ability. The scale mainly included 10 items, including eating, bathing, dressing, self-care of defecation and urination, toileting, bed to chair shifting, walking on level ground, and stair climbing, with a total of 25 items with a full score of 100 points. The higher the score, the stronger the self-care ability. (3) Quality of life questionnaire QLQ-H&N35 scale was used to evaluate the improvement effect of symptoms, including cough, pain, dry mouth, sticky saliva, dysphagia, and eating difficulty. The measurement time was 3 months after treatment; the lower the score was, the lighter the symptoms were. (4) The health survey short form SF-36 scale was used to evaluate the improvement effect of quality of life, including physiological function, role physical, physical pain, general health, energy, social function, emotional function, and mental health. The measurement time was 3 months after treatment; the higher the score, the better the quality of life. (5) Self-Rating Depression Scale (SDS) score and Self-Rating Anxiety Scale (SAS) score were used to evaluate the psychological state of the patients, and the measurement time was 3 months after treatment. SDS and SAS scores are as follows: less than 50 points indicates no depression/anxiety; a score of 50 to 60 indicates mild depression/anxiety; a score of >60 to 70 indicates moderate depression/anxiety. A score of >70 indicates severe depression/anxiety. (6) The mortality and disability rates of the two groups were observed during 2-year follow-up.

### 2.4. Statistical Analysis

SPSS 26.0 software was used for statistical analysis of data in this study. Measurement data were expressed by $\overset{¯}{x}\pm s$, and *t* test was used for the comparison between the two groups. The count data were expressed as rate (%) and were compared using *χ*^2^ test. *P* < 0.05 was considered statistically significant.

## 3. Results

### 3.1. Mini-Cog and MoCA Scores of the Two Groups of Patients

The Mini-Cog and MoCA scores of the patients in the research group were 26.24 and 27.82, respectively, showing significant differences (*P* < 0.05) compared with the 25.19 and 26.76 scores in the control group, as shown in Table 2.

### 3.2. The Self-Care Ability Scores of the Two Groups of Patients

Before radiotherapy, the self-care ability scores of the control group and the research group were 71.22 points and 70.16 points, and there was no significant difference between them (*P* > 0.05). After radiotherapy, the self-care ability score of patients in the research group was 76.89 points, significantly higher than 72.54 points in the control group (*P* < 0.05), as shown in Table 3.

### 3.3. Symptom Improvement Effect of Two Groups of Patients

The QLQ-H&N35 questionnaire scores of the patients in the research group were significantly lower than those in the control group in terms of cough, pain, dry mouth, sticky saliva, dysphagia, and eating difficulty (*P* < 0.05), as shown in Table 4.

### 3.4. The Improvement Effect of Quality of Life of the Two Groups of Patients

The scores of patients in the research group were higher than those in the control group in terms of physiological function, role physical, physical pain, general health, energy, social function, emotional function, and mental health, with significant differences (*P* < 0.05), as shown in Table 5.

### 3.5. Comparison of the SDS Score and SAS Score between Two Groups of Patients

The SDS score of the patients in the research group before radiotherapy was 76.62, and the SDS score of the patients in the control group before radiotherapy was 74.56. There was no significant difference between them (*P* > 0.05). After radiotherapy, the SDS scores of the patient in the research group and the control group were 58.18 and 66.39, respectively, showing significant differences (*P* < 0.05). Before radiotherapy, the SAS score of the patient in the research groups and the control groups was 71.60 and 72.89. There was no significant difference between them (*P* > 0.05). After radiotherapy, the SAS scores of the patient in the research group and the control group were 58.16 and 65.72, respectively, showing significant differences (*P* < 0.05), as shown in Table 6.

### 3.6. Comparison of the Mortality Rate between Two Groups of Patients

The mortality of the control group was higher than that of the research group, but the difference was not statistically significant (*P* > 0.05), as shown in Table 7.

## 4. Discussion

Brain glioma is a malignant tumor disease. At present, with the change of people's living habits, the incidence of brain glioma is increasing [12]. Although surgical resection of glioma lesions is the first choice in clinical practice, tumor cells grow in an infiltrative manner, and patients with surgery alone have a poor prognosis. Multiple adjuvant therapy methods are needed to further inhibit the malignant proliferation and metastasis of tumor cells.

Relevant studies [13] have shown that head and neck tumors are moderately sensitive to radiotherapy. Compared with conventional radiotherapy, three-dimensional conformal radiotherapy can avoid irradiation of 30% to 40% of normal brain tissue, thus effectively improving the local control rate of brain tumor and patient survival rate, and has become the first choice for brain tumor radiotherapy. Although it has good therapeutic effect, there are still problems such as incomplete target delineation and difficulty in meeting the uniformity of intensity, resulting in severe damage to peripheral lesions and affecting the quality of life of patients. Accurately delineating the target volume and adjusting the radiation dose are crucial for glioma patients [14, 15]. IMRT is an in vitro stereotactic radiotherapy developed on the basis of three-dimensional conformal radiotherapy, including photon beams, proton beams, and heavy ion beams. The method is based on the preoperative CT results of patients to develop targeted targets, and the targeted area is analyzed anatomically, and then, the intensity of radiation is adjusted to accurately deliver radiation to the lesions. It can not only increase the conformal degree of the target volume but also has the characteristics of scientific dose distribution, uniform dose in the radiation field, and compact dose gradient, which can effectively improve the tumor radiotherapy dose and reduce the radiation dose of normal tissues around the target volume, enhance the therapeutic effect, and improve the efficacy and safety of treatment [16]. Cancer patients have a series of psychological disorders due to the sudden knowledge of the disease and the worry about the disease in the hospital treatment process, the fear of bringing huge economic burden to the family, the fear of surgery, etc., which is not conducive to the postoperative rehabilitation of patients, affecting the quality of life of patients.

Quality of life is an indicator system that reflects the long-term impact of internal and external environment on human physiology, psychological, social activities, and life satisfaction. As an important part of the function of various organs, once the brain tissue is damaged, it will have a negative impact on the quality of life of patients. With the continuous development of diagnosis and treatment technology, as well as the continuous improvement of people's medical awareness, while focusing on the prognosis, more attention is paid to the quality of life of patients [17]. Improving the patient's quality of life means a positive change in both physical and psychological status, which is also a clinically accepted standard of prognosis. Therefore, how to improve the postoperative quality of life of patients through treatment is an important goal of intracranial tumor treatment [18]. In addition, most patients have a variety of nervous anxiety about the brain tumor, coupled with the various symptoms caused by the tumor, so that patients are prone to a variety of bad emotions during hospitalization, which have a negative impact on the prognosis of patients [19]. In addition to the highest dose of radiation irradiation at the primary tumor site, the surrounding adjacent tissues also inevitably received higher doses, leading to acute side reactions such as oral mucositis, oral pain, dry mouth, dysphagia, difficulty in opening the mouth, and decreased taste during radiotherapy [20]. Related studies suggest that there is a significant negative relationship between symptom severity and its quality of life in each time period before and after radiotherapy [21].

In this study, we found that the scores of self-care ability of patients who underwent three-dimensional conformal IMRT were significantly higher than those of the control group. In the results of the quality of life questionnaire, patients in the three-dimensional conformal IMRT research group had significantly less symptoms such as cough, pain, dry mouth, sticky saliva, dysphagia, and eating difficulty. This is because IMRT can protect the brain stem, spinal cord, and parotid gland, increase the conformal degree of target volume, and thus have a low impact on patients' normal self-care life and reduce the adverse reaction symptoms in the process of radiotherapy. It is well known that advanced radiation encephalopathy caused by radiation therapy can seriously affect the quality of life of patients. In our results, the improvement of quality of life in the research group was similar to the quality of life assessment results of children with brain tumor undergoing proton beam radiotherapy in Massachusetts General Hospital, USA, and the scores of 4 out of 5 assessment items in the proton beam radiotherapy group were similar to those in the healthy control group [22]. The research of M.D. Anderson Cancer Center also showed that proton beam radiotherapy is more beneficial to the protection of children's neurocognitive function and avoid intellectual impairment [23].

Due to the lack of understanding of the disease and the worry about treatment effect, cost, and other aspects, most patients with craniocerebral tumor have varying degrees of anxiety and depression, resulting in patients unable to actively cooperate with the treatment. Negative emotions also tend to lead to patients with reduced immunity, endocrine disorders, energy deficiency, and other serious impact on patients' quality of life. It affects the treatment and prognosis of patients [24]. Our study found that the scores of SDS and SAS of patients who underwent three-dimensional conformal IMRT were significantly lower than those of the control group. These results suggest that the negative emotions of patients in the research group have been improved.

This is consistent with our conclusion; namely, patients receiving three-dimensional conformal IMRT had higher Mini-Cog and MoCA scores, the scores of physiological functions, role physical, physical pain, general health, energy, social function, emotional function, and mental health were higher than those of the control group, and the negative effects on patients' functions were lower. Age and education had little effect on Mini-Cog. And it reduced the error caused by age and educational background [25]. The negative effects were due to irradiation of specific radiation-sensitive areas, such as the hippocampus, and the lasting effects of increased treatment. This is because the dose intensity and range of three-dimensional conformal IMRT are mainly adjusted according to the three-dimensional shape of the patient's target volume, the relationship between target volume and organ, and the anatomical relationship between target volume and organ, so as to avoid great damage to normal organs and tissues. These results suggest that controlling the dose of radiation to a specific target volume and uniform dose of irradiation can prevent brain injury and subsequent negative effects on patient's function. There was no significant difference in mortality between the two groups, possibly due to insufficient follow-up and the lower mortality rate of low-grade gliomas compared to high-grade gliomas.

In conclusion, three-dimensional conformal IMRT can delineate the target volume more accurately and regulate the radiation intensity, which has a positive effect on the improvement of symptoms and quality of life of patients with low-grade glioma, and is safe and effective.

## Figures and Tables

**Table 1:** Comparison of the general information of the two groups of patients.

Group	Cases	Age	Gender (male/female)
Control group	50	34.06 ± 5.81	26.76 ± 2.02
Research group	50	38.63 ± 8.21	27.82 ± 1.43
*T* value		1.671	2.018
*P* value		0.831	0.994

**Table 2:** Comparison of Mini-Cog and Mo CA scores between the two groups of patients ($\overset{¯}{x}\pm s$, points).

Group	Cases	Mini-Cog	MoCA
Control group	50	5.46 ± 0.76	26.76 ± 2.02
Research group	50	7.59 ± 0.83	27.82 ± 1.43
*T* value		-1.083	-3.028
*P* value		0.001	0.003

**Table 3:** Comparison of self-care ability scores between the two groups of patients ($\overset{¯}{x}\pm s$, points).

Group	Cases	Before radiotherapy	After radiotherapy
Control group	50	71.22 ± 12.23	72.54 ± 7.69
Research group	50	70.16 ± 15.12	76.89 ± 9.87
*T* value		0.385	-2.458
*P* value		0.701	0.016

**Table 4:** Comparison of symptom improvement effect between two groups of patients ($\overset{¯}{x}\pm s$, points).

Group	Cases	Cough	Pain	Dry mouth	Sticky saliva	Dysphagia	Eating difficulty
Control group	50	1.21 ± 0.30	4.24 ± 0.87	2.25 ± 0.48	1.25 ± 0.22	5.65 ± 1.27	2.05 ± 0.38
Research group	50	0.91 ± 0.23	4.03 ± 0.62	1.86 ± 0.39	1.03 ± 0.31	4.79 ± 1.12	1.95 ± 0.51
*T* value		3.741	2.603	3.316	2.232	3.591	1.112
*P* value		0.001	0.011	0.001	0.028	0.001	0.269

**(a):** 

Group	Cases	Physiological function	Role physical	Physical pain	General health
Control group	50	84.34 ± 5.12	72.12 ± 6.33	73.76 ± 7.45	73.87 ± 8.45
Research group	50	87.41 ± 7.34	76.37 ± 7.12	78.41 ± 9.19	77.56 ± 7.04
*T* value		-2.426	-3.154	-2.779	-2.372
*P* value		0.017	0.002	0.007	0.020

**(b):** 

Group	Cases	Energy	Social function	Emotional function	Mental health
Control group	50	66.67 ± 7.88	79.54 ± 9.03	82.56 ± 6.31	81.56 ± 6.78
Research group	50	71.12 ± 7.81	86.11 ± 8.23	85.77 ± 5.92	85.72 ± 7.01
*T* value		-2.836	-3.082	-2.623	-3.061
*P* value		0.006	0.001	0.010	0.003

**Table 6:** Comparison of the SDS score and SAS score between two groups of patients ($\overset{¯}{x}\pm s$, points).

Group	Cases	SDS score before radiotherapy	SDS score after radiotherapy	SAS score before radiotherapy	SAS score after radiotherapy
Control group	50	74.56 ± 5.12	66.39 ± 6.18	72.89 ± 6.53	65.72 ± 5.50
Research group	50	76.62 ± 5.94	58.18 ± 5.84	71.60 ± 5.98	58.16 ± 7.52
*T* value		1.204	8.206	0.840	8.682
*P* value		0.207	<0.001	0.873	0.006

**Table 7:** Comparison of the mortality rate between two groups of patients (*n*, %).

Group	Cases	Death
Control group	50	2 (4%)
Research group	50	1 (2%)
*X* ^2^ value		4.321
*P* value		0.701

## Data Availability

The labeled datasets used to support the findings of this study are available from the corresponding author upon request.
